The article "Diseases That Occur Prior to Spontaneous Intracerebral Hemorrhage: Identification of Predisposing and Risk Factors Using Lag Sequential Analysis" was published in 2022. Journal: J Healthc Eng.

# Diseases That Occur Prior to Spontaneous Intracerebral Hemorrhage: Identification of Predisposing and Risk Factors Using Lag Sequential Analysis

**DOI:** 10.1155/2022/9733712

**Published:** 2022-03-25

**Authors:** Hsien-Wei Ting, Ting-Ying Chien, Chun-Chih Liao

**Affiliations:** ^1^Department of Neurosurgery, Taipei Hospital, Ministry of Health and Welfare, New Taipei City, Taiwan; ^2^Graduate Program in Biomedical Informatics, Yuan Ze University, Taoyuan City, Taiwan; ^3^Department of Computer Science and Engineering, Yuan Ze University, Taoyuan City, Taiwan; ^4^Innovation Center for Big Data and Digital Convergence, Yuan Ze University, Taoyuan City, Taiwan; ^5^Institute of Biomedical Engineering, National Taiwan University, Taipei City, Taiwan

## Abstract

Spontaneous intracerebral hemorrhage (sICH) has many predisposing/risk factors. Lag sequential analysis (LSA) is a method of analyzing sequential patterns and their associations within categorical data in different system states. The results of this study will assist in preventing sICH and improving the patient outcome after sICH. The correlations between a first sICH and previous clinic visits were examined using LSA with data obtained from the Taiwan National Health Insurance Research Database (NHIRD). In this study, LSA was employed to examine the data in the Taiwan NHIRD in order to identify predisposing and risk factors related to sICH, and the results increased our knowledge of the temporal relationships between diseases. This study employed LSA to identify predisposing/risk factors prior to the first occurrence of sICH using a healthcare administrative database in Taiwan. The data were managed using the clinical classification software (CCS). All cases of traumatic ICH were excluded. Ten disease groups were identified using CCS. Hypertension and dizziness/vertigo were identified as two important predisposing/risk factors for sICH, and early treatment of hypertension resulted in a greater survival rate. Five disease groups were found to have occurred prior to other diseases and affected mostly the elderly, resulting in subsequent sICH. The results of this study also showed that nutritional status and tooth health were highly associated with the occurrence of sICH owing to a poor state of the digestive system. In conclusion, there are many diseases that influence the risk of a subsequent sICH. This study demonstrated that LSA is a very useful tool for future study of healthcare administrative databases.

## 1. Background

Spontaneous intracerebral hemorrhage (sICH) is an important disease and carries a relatively high mortality and morbidity [1–4]. The early and properly aggressive care are needed, and these patients cost a lot of medical expenditures [3–5]. Although there are relative medical diseases, the surgical intervention for sICH patients is needed [4]. Increased knowledge of the risk factors related to sICH will improve the prognosis of patients [6]. There are many predisposing and risk factors, including older age, gender, air pollution, climate, rural/urban location, alcohol consumption, hyperlipidemia, smoking, and drugs abuse and some chronic conditions [1, 3, 6–11]. The most important risk factor for sICH is hypertension [3, 11], while chronic kidney disease is highly correlated with ischemic stroke [12]. Antiplatelet agents, used for the prevention of the ischemic stroke, will increase the bleed volume of sICH and caused the worse clinical outcome [3]. Knowing and preventing the risk factors and predispose factors of sICH are the basic works. However, the subsequent occurrence of sICH in patients who possess the identified risk factors and the short-term risk factors are as yet unknown.

The article "Diseases That Occur Prior to Spontaneous Intracerebral Hemorrhage: Identification of Predisposing and Risk Factors Using Lag Sequential Analysis" was published in 2022. Journal: J Healthc Eng.

Lag sequential analysis (LSA) was proposed by Bakeman in 1978 and is a method of analyzing sequential patterns of categorical data represented in different system states [13–15]. LSA is suitable for finding the significant transition of a single event. Unlike time sequence analysis, LSA is more suitable for unbalanced data. LSA has been used widely in the detection of patterns of behaviors or behavioral changes of subjects of differing status, such as given behaviors, conditional behaviors, and some lag behaviors [15]. LSA can be employed to evaluate sequential patterns and their associations with observed and expected probabilities [14]. It has been used in many different research fields, in particular for behavioral observation of normal subjects, psychiatric patients, children, and athletes [14–20]. LSA has also been applied to support problem-solving and decision-making in the airport security screening process [21]. It can also be used to evaluate the actions of verbal and nonverbal communication of patients with depression during treatment [17]. LSA allows evaluation of categorical data in five fields: event sequence data, state sequence data, timed state sequence data, interval sequence data, and multievent sequence data [15]. This study employed LSA to identify predisposing/risk factors that are present prior to the first occurrence of sICH using data of patients included in the healthcare administrative database in Taiwan. The results of this study will assist in preventing sICH and improving the patient outcome after sICH.

## 2. Materials and Methods

The Taiwan National Health Insurance Research Database (NHIRD) is a medical electronic administrative database that contains both out-patient and hospital admission data and can be linked to government-issued open data and other research datasets. The NHIRD covers more than 99.6% of the Taiwanese population with all data of the clinics/hospitals seeking and administrative data [22]. The advantage of the NHIRD is that patient administrative data are collected longitudinally; this then enables evaluation of both predisposing and risk factors prior to the occurrence of diseases [8, 9, 23]. This study used NHIRD from 2006 to 2010 [22]. All first-occurrence sICH patients were included, with sICH defined according to International Classification of Diseases Ninth Revision (ICD-9) code 431 and totaling 2088 cases. Intracranial hemorrhage patients who were admitted due to a traumatic cause (ICD-9 codes 800.00–804.99, 850.00–854.19, 959.01, and 959.09) (52 cases) were excluded in this study, resulting in a final study sample of 2036 patients who suffered first sICH. This study was approved by the Institutional Review Board (IRB) of Taipei Hospital (IRB Approval Number: TH-IRB-0015-0003). A flowchart of data management is shown in Figure 1.

The article "Diseases That Occur Prior to Spontaneous Intracerebral Hemorrhage: Identification of Predisposing and Risk Factors Using Lag Sequential Analysis" was published in 2022. Journal: J Healthc Eng.

Diseases were defined according to the single-level clinical classification software (CCS) procedure category. Patients' medical profiles upon hospital admission and information regarding diseases suffered prior to the first sICH were collected. The Student *t*-test was used for continuous data, and standard deviations (SDs) were also calculated. The *χ*^2^ test was used for categorical data. SPSS version 24.0 (SPSS Inc., Chicago, IL, USA) was employed for demographic data analysis. Statistical significance was defined as *P* < 0.001. This study also employed a web-based tool [24] to carry out LSA, and the *Z* test significance from LSA was defined as *P* < 0.001.

## 3. Results

In total, 2036 patients (male/female = 1264/772) were included in this study. The mean age was 63.0 years (SD = 15.0), and the mean ages of the male and female patients were 60.6 years (SD = 14.5) and 66.9 years (SD = 15.0), respectively (*P* < 0.001). The mean survival duration was 2.9 years (SD = 2.3); this did not differ significantly between the male (3.0 years, SD = 2.3) and female patients (2.9 years, SD = 2.2). The admission fee following a first sICH was US$ 7441 (SD = 12476), and there was no significant difference between the male (US$ 7561, SD = 12456) and female patients (US$ 7245, SD = 12516). The mean length of stay and ICU length of stay were 30.8 days (SD = 66.0) and 7.7 days (SD = 12.9), respectively, and there was no significant difference in either duration between the male (31.8 days, SD = 65.7; 7.7 days, SD = 13.9) and female patients (29.2 days, SD = 66.6; 7.8 days, SD = 11.0). On average, the patients experienced 19.1 (SD = 10.3) diseases prior to the first sICH, and the mean number of diseases in the female patients (22.3 diseases, SD = 10.6) was significantly higher than in the male patients (17.1 diseases, SD = 9.6) (*P* < 0.001). The mortality rate within 30 days and within one year was 19.8% and 29.3%, respectively, and there were no significant differences in these mortality rates between the male (19.1% and 28.2%) and female patients (21.0% and 31.2%). The definition of a prolonged ICU stay was 10 days [2], and according to this definition, 26.5% of patients admitted for a first sICH had a prolonged ICU stay; there was no significant difference in this percentage between the male (26.2%) and female patients (26.9%) (Table 1).

The article "Diseases That Occur Prior to Spontaneous Intracerebral Hemorrhage: Identification of Predisposing and Risk Factors Using Lag Sequential Analysis" was published in 2022. Journal: J Healthc Eng.

LSA performed to analyze the mean durations between the first occurrences of diseases and the first sICH were evaluated. Ten significant disease groups according to the CCS were identified by lag sequential analysis (LSA): inflammation/infection of the eye (except when caused by tuberculosis or a sexually transmitted disease) (CCS090; 39.6 months, SD = 45.0); conditions associated with dizziness or vertigo (CCS093; 27.9 months, SD = 40.5); essential hypertension (CCS098; 42.0 months, SD = 46.9); acute bronchitis (CCS125; 35.3 months, SD = 43.7); other upper respiratory infections (CCS126; 79.6 months, SD = 41.7); disorders of the teeth and jaw (CCS136; 80.9 months, SD = 58.3); gastritis and duodenitis (CCS140; 26.3 months, SD = 40.6); other nontraumatic joint disorders (CCS204; 32.0 months, SD = 42.9); spondylosis, intervertebral disc disorders, other back problems (CCS205; 46.8 months, SD = 46.6); and other connective tissue diseases (CCS211; 43.3 months, SD = 46.5) (Table 2).

A total influence flowchart is shown in Figure 2. In general, the CCS diseases group that was most highly correlated with a subsequent first sICH in patients who had visited the clinic was “conditions associated with dizziness or vertigo (CCS093),” with a *Z* score of 8.222, followed by “essential hypertension (CCS098),” *Z* score 5.440; “inflammation or infection of the eye (except when caused by tuberculosis or a sexually transmitted disease) (CCS090),” *Z* score 5.395; “gastritis and duodenitis (CCS140),” *Z* score 4.098; and “other nontraumatic joint disorders (CCS204),” *Z* score 3.682. Most paths originated from CCS136, “disorders of the teeth and jaw;” the first path was from CCS136 to CCS098, “essential hypertension” (*Z* score = 4.799), and then to the occurrence of a first sICH. The second path was from CCS136 to CCS126, “other upper respiratory infections” (*Z* score = 23.316), then to CCS090, “inflammation or infection of the eye (except when caused by tuberculosis or a sexually transmitted disease)” (*Z* score = 5.642), and then to a first sICH. Another path was from CCS126 “other upper respiratory infections” to CCS205 “spondylosis, intervertebral disc disorders, other back problems” (*Z* score = 4.147), CCS125 “acute bronchitis” (*Z* score = 6.818), and CCS204 “other nontraumatic joint disorders” (*Z* score = 4.989). CCS204 “other nontraumatic joint disorders” may have a direct path to the first occurrence of sICH or may be pathed to CCS093 “conditions associated with dizziness or vertigo” (*Z* score = 3.185) and then to first sICH. A short path was from CCS211 “other connective tissue diseases” to CCS093 “conditions associated with dizziness or vertigo” (*Z* score = 3.292) and then to the first sICH (Figure 2).

The article "Diseases That Occur Prior to Spontaneous Intracerebral Hemorrhage: Identification of Predisposing and Risk Factors Using Lag Sequential Analysis" was published in 2022. Journal: J Healthc Eng.

When examining the patients who had died within 30 days, only CCS090 “inflammation and infection of the eye (except when caused by tuberculosis or a sexually transmitted disease)” had a path to a first sICH, with a *Z* score of 3.568; the other aforementioned relationships disappeared (Figure 3). Within the group of patients who were alive after 30 days, four disease/condition groups remained significant: CCS093 “conditions associated with dizziness or vertigo” (*Z* score = 7.763); CCS098 “essential hypertension” (*Z* score = 5.443); CCS090 “inflammation or infection of the eye (except when caused by tuberculosis or a sexually transmitted disease)” (*Z* score = 4.273); and CCS140 “gastritis and duodenitis” (*Z* score = 3.394). CCS204 “other nontraumatic joint disorders” was not significantly correlated with a subsequent first sICH. The initial disease was CCS136 “disorders of the teeth and jaw;” a clinic visit for CCS136 “disorders of teeth and jaw” was correlated with subsequent CCS098 “essential hypertension” (*Z* score = 3.602); CCS126 “other upper respiratory infections” (*Z* score = 21.392); and CCS205 “other back problems” (*Z* score = 3.304). CCS126 had a path to CCS090 (*Z* score = 5.685), then a path to first sICH, but CCS205 “other back problems” pathed to CCS204 “other nontraumatic joint disorders,” while CCS204 “other nontraumatic joint disorders” did not path to sICH if the patient remained alive within 30 days of sICH (Figure 4).

Examining the sICH patients who died within one year of sICH occurrence, the paths were found to be simpler. CCS125 “acute bronchitis” was not significantly correlated with these sICH patients. CCS93 “conditions associated with dizziness or vertigo” (*Z* score = 3.324) and CCS140 “gastritis and duodenitis” (*Z* score = 3.455) had direct paths to sICH in the patients who died within one year. CCS136 “disorders of the teeth and jaw” was the initial point of the pathway, to CCS098 “essential hypertension” (*Z* score = 3.733) and then CCA126 “other upper respiratory infections” (*Z* score = 3.310), or via a direct path to CCS126 “other upper respiratory infections” (*Z* score = 11.786). CCS126 “other upper respiratory infections” then pathed in two directions: CCS090 “inflammation or infection of the eye (except when caused by tuberculosis or a sexually transmitted disease)” (*Z* score = 3.314) and CCS204 “other nontraumatic joint disorders” (*Z* score = 3.131). These then pathed to sICH in the patients who died within one year, with a *Z* score of 3.386 and 3.378, respectively (Figure 5). In the sICH patients who were alive after one year (Figure 6), CCS125 “acute bronchitis,” CCS140 “gastritis and duodenitis,” CCS204 “other nontraumatic joint disorders,” and CCS205 “other back problems” were not significantly correlated with sICH. CCS098 “essential hypertension” (*Z* score = 4.974) and CCS093 “conditions associated with dizziness or vertigo” (*Z* score = 7.666) directly influenced the sICH patients who were alive after one year, and CCS126 “other upper respiratory infections” influenced these two categories of disease (*Z* score = 3.535/4.584). CCS136 “disorders of the teeth and jaw” influenced CCS098 “essential hypertension” (*Z* score = 3.300) and CCS126 “other upper respiratory infections” (*Z* score = 20.147).

The article "Diseases That Occur Prior to Spontaneous Intracerebral Hemorrhage: Identification of Predisposing and Risk Factors Using Lag Sequential Analysis" was published in 2022. Journal: J Healthc Eng.

## 4. Discussion

LSA is a method used for behavior evaluation, such as patterns of behaviors or behavioral change [15]. LSA is also employed to evaluate sequential and lag patterns of subjects with probabilities [14]. The Taiwan NHIRD contains longitudinal data, which have been used to support many epidemiology studies in different fields [1, 2, 8, 9, 22, 23, 25, 26]. Recently, manifestations of the longitudinal data in the NHIRD were found. This study used LSA, a longitudinal data analysis method, with data from the NHIRD to identify predisposing and risk factors for a first sICH. Other longitudinal data analysis methods have been used in conjunction with the NHIRD to increase our knowledge of the relationships between diseases with time [26, 27]; this represents a key area of the future study of medical administrative databases.

The major risk factors for stroke are aging, hypertension, diabetes mellitus, hyperlipidemia, obesity, tobacco smoking, and poor diet/nutrition [1, 26, 28]. This study focused on the risk factors of patients who had visited the clinic previously. It is very logical that hypertension (CCS_0098) is identified at a clinic visit prior to the occurrence of sICH. Conditions associated with dizziness or vertigo (CCS_0093) were also identified as being important in clinic visits prior to the first occurrence of sICH, and it was second longer time period from the first visit to the clinics for this reason to the sICH attacked. It is possible that poor control of blood pressure identified at a clinic visit could cause dizziness and vertigo, and it might be that the patient is first found to have prehypertension. Hypertension and dizziness/vertigo were the two most important predisposing/risk factors in first-occurrence sICH patients who were alive after 30 days, and in the sICH patients who died within 30 days, the only prior disease/symptom group was dizziness and vertigo. This may be because these patients had been diagnosed with hypertension but had poor control of their blood pressure, which causes severe damage after sICH. Alternatively, although they have experienced sICH, patients with an early diagnosis of high blood pressure (at a previous clinic visit) and better control of their blood pressure will have a better outcome. In this study, no other prior disease/symptom groups were identified as being correlated with the first occurrence of sICH, such as, for example, diabetes or hyperlipidemia. The manifestations of predisposing and risk factors differ between patients with sICH and those with ischemic stroke [12].

The article "Diseases That Occur Prior to Spontaneous Intracerebral Hemorrhage: Identification of Predisposing and Risk Factors Using Lag Sequential Analysis" was published in 2022. Journal: J Healthc Eng.

Previous studies have shown that aging is one of the most important risk factors for stroke, especially sICH [1, 2, 26, 29–31]. Three aging-related disease groups were examined in this study: other nontraumatic joint disorders (CCS_0204), spondylosis, intervertebral disc disorders, and other back problems (CCS_0205), and other connective tissue diseases (CCS_0211). Most elderly patients will have these conditions. Our analysis highlighted some interesting results, in which these three diseases were conditions that occurred prior to other diseases, in the same way that acute bronchitis (CCS_0125) and other upper respiratory infections (CCS_0126) were both found to occur prior to other diseases, and the patients visiting clinics and suffering sICH will be mostly elderly. Airway infections also influence other diseases and consequently sICH, COVID-19 being a good example of this. The mortality and morbidity rates in the elderly are significantly higher than in younger patients [32]. These diseases are important aging-related diseases and will worsen the condition of patients both before and after sICH.

Studies have shown that nutritional status and tooth health are highly associated with the outcome of stroke patients [30, 33]. There were no significantly different findings between the sICH patients who died and who were alive no matter after 30 days or after a year, with the exception of the occurrence of disorders of the teeth and jaw (CCS_0136). However, there was a longer duration between the occurrence of CCS_0136 in patients and first sICH, and this result provided indirect evidence of the importance of nutrition and tooth health. These patients will suffer malnutrition and other diseases prior to sICH. Tooth health will influence the nutrition of elderly patients, and as a consequence, the mortality of first-occurrence sICH patients. Clinic visits for gastritis and duodenitis (CCS_0140) had a similar but more direct consequence, and the duration between those visits and the first sICH was shorter than for other diseases (26.3 months, SD = 40.6). Fortunately, gastritis and duodenitis were no longer of influence in subsequent first-occurrence sICH patients who remained alive for more than one year. This result indirectly proved the importance of gastrointestinal function and nutrition.

The article "Diseases That Occur Prior to Spontaneous Intracerebral Hemorrhage: Identification of Predisposing and Risk Factors Using Lag Sequential Analysis" was published in 2022. Journal: J Healthc Eng.

It is very surprising that we found that diseases involving infection or inflammation of the eye commonly occurred prior to a first sICH, and this disease group influenced the first sICH very directly. There have been no reports of correlations between inflammation or infection of the eye and sICH; however, stroke patients often have some neuroophthalmic manifestations, such as ocular motility abnormalities, visual acuity, and visual field defects [34]. These might be first treated as eye inflammation or infection when patients visit the clinic or may simply be considered aging-related diseases. The correlations between sICH and infection or inflammation of the eye require further study.

There were some limitations of this study. First, this study used the first clinic visit as the data obtained from the Taiwan NHIRD. This study was an example of the sequential study of diseases. We did not evaluate the details of all clinic visits owing to them not being convergent in the study. In the future, we may study the NHIRD in more detail. Second, this study only evaluated sICH using a medical administrative database; the data did not include behavioral information and data on the medical treatment of stroke patients. The sICH patients in this study also did not include these data. We may study all stroke patients in other databases that include more detailed data in the future. Third, some results of this study have not been discussed previously in the literature and hence provide a good platform for further study. The results could then be taken into account to inform disease prevention and surveillance.

## 5. Conclusion

It is important for the future study to analyze medical administrative databases using suitable tools. This study employed LSA to analyze data contained in the Taiwan NHIRD in order to identify predisposing and risk factors for sICH and to increase knowledge of the relationships between diseases with time. Hypertension and dizziness/vertigo were identified in this study as two important predisposing/risk factors for sICH. Early treatment of hypertension resulted in a better survival rate. The results demonstrated that five disease groups occurred prior to other diseases and mostly affected elderly patients, with the consequence of sICH. The study results also indicated that nutritional status and tooth health were highly associated with the first occurrence of sICH due to poor functioning of the digestive system. In conclusion, there are many prior diseases that influence subsequent sICH.

The article "Diseases That Occur Prior to Spontaneous Intracerebral Hemorrhage: Identification of Predisposing and Risk Factors Using Lag Sequential Analysis" was published in 2022. Journal: J Healthc Eng.

## Figures and Tables

**Figure 1:** Flowchart of data management. NHIRD, National Health Insurance Research Database, 2006–2010. sICH ICD-9 code 431: 2,088 cases in total. Cases of suspected traumatic ICH (ICD-9 codes 800.00–804.99, 850.00–854.19, 959.01, and 959.09) were excluded in this study, resulting in 2036 cases remaining for analysis.

**Figure 2:** Disease transition diagram to first-occurrence sICH (all patients).

**Figure 3:** Disease transition diagram to first-occurrence sICH (patients who died within 30 days of sICH).

**Figure 4:** Disease transition diagram to first-occurrence sICH (patients who were alive 30 days after sICH).

**Figure 5:** Disease transition diagram to first-occurrence sICH (patients who died within one year of sICH).

**Figure 6:** Disease transition diagram to first-occurrence sICH (patients who were alive one year after sICH).

**Table 1:** Demographic data of the sICH patients.

	Male	Female	Total
Case number (*N*)	1264	772	2036
Mean age (years) (SD)^*∗∗∗*^	60.6 (14.5)	66.9 (15.0)	63.0 (15.0)
Survival duration (years) (SD)	3.0 (2.3)	2.9 (2.2)	2.9 (2.3)
Admission fee (SD)	7561 (12456)	7245 (12516)	7441 (12476)
Length of hospital stay (SD)	31.8 (65.7)	29.2 (66.6)	30.8 (66.0)
ICU length of stay (SD)	7.7 (13.9)	7.8 (11.0)	7.7 (12.9)
Mean number of diseases at clinic visits (SD)^*∗∗∗*^	17.1 (9.6)	22.3 (10.6)	19.1 (10.3)
Monthly death rate (%)	19.1	21.0	19.8
Yearly death rate (%)	28.2	31.2	29.3
Prolonged ICU stay rate (%)	26.2	26.9	26.5

^*∗∗∗*^Statistically significant, *P* < 0.01. SD, standard deviation.

**Table 2:** List of disease groups prior to sICH, incidence, and duration from first clinic visit to first sICH (months).

CCS	Disease group	Alive (%)	Dead (%)	Total (%)	Time period^$^ (SD)
CCS_0090^#^	Inflammation/infection of the eye	53.3	51.9	53.0	39.6 (45.0)
CCS_0093	Conditions associated with dizziness or vertigo	43.4	45.4	43.8	27.9 (40.5)
CCS_0098	Essential hypertension	57.1	59.3	57.6	42.0 (46.9)
CCS_0125	Acute bronchitis	48.7	47.1	48.4	35.3 (43.7)
CCS_0126	Other upper respiratory infections	87.4	86.1	87.2	79.6 (41.7)
CCS_0136^*∗*^	Disorders of the teeth and jaw	75.6	70.5	74.6	80.9 (58.3)
CCS_0140	Gastritis and duodenitis	37.5	39.0	37.8	26.3 (40.6)
CCS_0204	Other nontraumatic joint disorders	43.8	47.1	44.5	32.0 (42.9)
CCS_0205	Spondylosis, intervertebral disc disorders, and other back problems	61.7	60.5	61.4	46.8 (46.6)
CCS_0211	Other connective tissue diseases	57.1	59.6	57.6	43.3 (46.5)

^#^Except when caused by tuberculosis or a sexually transmitted disease. ^*∗*^*P* < 0.05, significant difference between the patients who were alive and those who died no matter 30 days or one year. ^$^Mean months and standard deviation (SD).

The article "Diseases That Occur Prior to Spontaneous Intracerebral Hemorrhage: Identification of Predisposing and Risk Factors Using Lag Sequential Analysis" was published in 2022. Journal: J Healthc Eng.

## Data Availability

The datasets used to support the findings of this study are available from the National Health Insurance Administration, NHRI, Taiwan.
